The article "Analysis on the Efficacy of Bronchial Artery Chemoembolization Combined with 125I Seed Implantation in the Therapy of Advanced Non-Small-Cell Lung Cancer Based on the Medical Database" was retracted in 2023. Reasons: signs of a paper mill; compromised peer review; unreliable results or conclusions.

# Analysis on the Efficacy of Bronchial Artery Chemoembolization Combined with 125I Seed Implantation in the Therapy of Advanced Non-Small-Cell Lung Cancer Based on the Medical Database

**DOI:** 10.1155/2022/7376844

**Published:** 2022-06-24

**Authors:** Peng Xie, Lidong He, Yan Zhang

**Affiliations:** ^1^Sixth Medical Center of PLA General Hospital, Beijing 100048, China; ^2^China-Japan Friendship Hospital, Beijing 100048, China

## Abstract

**Objective:**

To investigate the use and the efficacy of bronchial artery chemoembolization combined with 125I seed implantation in advanced non-small-cell lung cancer (NSCLC) therapy based on the medical database.

**Methods:**

A total of 102 patients with advanced NSCLC were randomly divided into two groups. The control group was treated with 125I seed implantation, and the observation group was treated with bronchial artery chemoembolization (BACE) combined with 125I seed implantation based on medical database. The clinical efficacy, carcinoembryonic antigen (CEA), cytokeratin 19 fragment antigen 21-1 (CYFRA21-1), glycan antigen 125 (CA125), peripheral blood CD3+, CD8+, CD4+/CD8+ T cells, insulin-like growth factor type 1 receptor (IGF-1R), S100 calcium-binding protein A2 (S100A2), long-term efficacy (time to disease progression, six-month survival rate, and one-year survival rate), and safety were then analyzed.

**Result:**

The disease remission rate in the observation group was 62.75%, which was higher than that in the control group (41.18%). After 1 month and 3 months of treatment, the levels of serum CYFRA21-1, CEA, CA125, and IGF-1R were lower, while serum S100A2 was higher in the observation group than in the control group (*P* < 0.05). For safety assessment, we found that the incidences of neutropenia, thrombocytopenia, and gastrointestinal reactions had no statistical differences between two groups. The time to disease progression in the observation group was 129.85 d longer than that in the control group, 89.74 d, and the six-month survival rate and 1-year survival rate were higher in the observation group relative to the control group.

**Conclusion:**

Medical database-based BACE combined with 125I seed implantation in the therapy of advanced NSCLC patients has definite efficacy with certain safety, which can enhance antitumor effect and prolong survival rate in advanced NSCLC patients.

## 1. Introduction

Non-small-cell lung cancer (NSCLC) is the main type of primary lung cancer, accounting for about 85% of all lung cancer cases. Most of the patients have developed to the middle or advanced stage when they were first diagnosed, leading to the loss of the best opportunity for surgery [1]. In recent years, minimally invasive treatment methods such as cryotherapy, particle implantation, radio frequency, and microwave have been gradually applied in clinic [2]. Continuous low-dose-rate radiotherapy with 125I seed implantation can significantly improve the lethality for tumor cells and simultaneously protect surrounding normal tissues, with less trauma and fewer complications; importantly, the use of it has achieved remarkable results in local control and palliative treatment in lung cancer, prostate cancer, and pancreatic cancer [3]. Bronchial artery chemoembolization (BACE) is one of the significant technologies for the palliative therapy in lung cancer, antitumor drugs are injected into the lesions through microcatheters, and embolization materials are used to block the blood vessels of the lesions to achieve the purpose of killing tumor cells [4].

Therefore, we attempted to uncover the clinical value of the application of BACE combined with 125I seed implantation based on medical database in advanced NSCLC treatment, which may be beneficial to NSCLC effective treatment.

## 2. Materials and Methods

### 2.1. Clinical Patients

A total of 102 patients with advanced NSCLC were collected in our hospital from January 2019 to August 2020 and randomly divided into two groups of 51 cases each. All patients were histologically diagnosed as NSCLC at stage IIIb/IV that had missed opportunities for surgery. None of them had undergone preoperative treatment, and the estimated survival time of all participates was longer than 6 months. Among them, 57 cases were male, and the rest was female (*n* = 45); the age ranged from 38 to 85 years, with an average of 62.79 ± 10.55 years. The exclusion criteria included those with visible cavity in the tumor, those with a distance from the tumor to the great blood vessels ≤ 0.5 cm, those with other acute or chronic serious diseases, and those who have recently used anticoagulant drugs. The clinicopathological features of 102 NSCLC patients are shown in Table 1. All patients had provided written informed consent, and the study was approved by the Ethics Committee of our hospital.

### 2.2. Treatment

After admission, a cisplatin and vinorelbine (NP) regimen was adopted: 25 mg/m^2^ vinorelbine was intravenously injected on the 1st and 8th days; 25 mg/m^2^ cisplatin was intravenously injected on the 1st to 3rd days; 28 days were one cycle, with a total of 2 cycles. At the same time, two groups of the following treatments were given:

1. *Control group*: 125I seed implantation. The patient was placed in the supine position, and CT scanning was performed to locate the upper and lower boundaries of the tumor and the extent of the tumor area. Combined with the radioactive particle therapy planning system (TPS), the patient's body surface was marked. Routine skin disinfection, 2% lidocaine infiltration anesthesia, needle insertion angle and level according to TPS, adjusting the needle insertion depth and angle under CT scan until the seed implantation needle reaches the distal end of the tumor. Using the needle withdrawal method, each particle was placed in the tumor one by one using a particle implantation gun, and the particle distribution was required to be consistent with the preoperative plan. After seed implantation, CT scan was performed again to observe the occurrence of hemothorax, pneumothorax, and particle displacement; the images were input into the TPS system to verify the particle dose, and dose cooling was performed on the day of surgery or within 1 week after surgery; district particle reseeding
2. *Observation group*: BACE combined with 125I seed implantation. On the basis of the above, BACE based on medical database was performed, one side of the artery was punctured and intubated under local anesthesia, and a 5 F angiography catheter was placed for angiography to observe the course of the bronchial artery and the blood supply to the tumor. The perfusion range includes tumor foci, involved lymph nodes in the mediastinum, and bronchial arteries, avoiding the intercostal arteries, and does not block blood flow during perfusion. After confirmation by microcatheter superselective angiography, cisplatin 75 mg/m^2^ and gemcitabine 1000 mg/m^2^ were injected through the catheter. After perfusion, microsphere embolization particles (Embosphere, 300-500 *μ*m, 560-710 *μ*m) and gelatin sponge were used to embolize the target vessel to occlude; postoperative routine antiemetic and hydration; 1 time/4 weeks, 3 times/course

### 2.3. Observation of Indicators

1. *Clinical efficacy*: according to the WHO 1981 standard, complete remission: complete focus debridement; partial remission: lesion reduction ≥ 50%, but incomplete absorption; stable: the lesion increases ≤25% or decreases <50%; progress: the foci expanded by 25%. Disease remission rate is the percentage of total remission and partial remission

The blood samples from all patients were collected before treatment, 1 month after treatment, and 3 months after treatment.

(2) *Tumor markers*: the blood was centrifuged at 3500 r/min for 10 min, and then, the sera were collected to detect the levels of carcinoembryonic antigen (CEA) and carbohydrate antigen 125 (CA125) by radioimmunoassay or cytokeratin 19 fragment antigen 21-1 (CYFRA21-1) by electrochemical assay using corresponding commercial kit (Mlbio, Shanghai, China) according to the kit instructions
(3) *Peripheral blood T lymphocyte subsets*: 5 ml peripheral blood was placed in an anticoagulation tube, and then, the EPICSXL flow cytometer (Beckman Coulter, USA) was applied to assay the changes of T lymphocyte subsets CD3+, CD8+, and CD4+/CD8+
(4) *Serum indicators*: the blood of patients was centrifuged at 3500 r/min for 10 min to obtain the sera. Thereafter, levels of insulin-like growth factor type 1 receptor (IGF-1R) and S100 calcium-binding protein A2 (S100A2) were determined by ELISA as per the protocol of corresponding commercial kits (Mlbio)
(5) *Long-term efficacy*: follow-up for 1 year, the time of disease progression, half-year survival rate, and 1-year survival rate of the two groups were calculated
(6) *Safety*: the toxic and side effects of antitumor drugs are classified into grades 0-IV according to WHO standards, including neutropenia, thrombocytopenia, and gastrointestinal reactions

### 2.4. Statistical Analysis

Statistical analyses were performed by SPSS 23.0. Measurement data were manifested by mean ± standard deviation (SD), and enumeration data were expressed by *n* (%). The differences between groups were assessed by Student's *t*-test or *χ*^2^ test. *P* value < 0.05 implied statistically significant.

## 3. Results

### 3.1. Clinical Characteristics in Patients with Advanced NSCLC

As displayed in Table 2, there was no statistical difference in gender, age, pathological classification, clinical stage, and medical payment method between the observation group and the control group (*P* > 0.05).

### 3.2. Clinical Efficacy between the Two Groups

As shown in Table 3, the disease remission rate in the observation group was 62.75% which was significantly higher than that in the control group (41.18%) (*P* < 0.05).

### 3.3. Comparison of Tumor Markers between the Two Groups

Before treatment, there was no difference in observation group and the control group in the levels of CEA, CYFRA21-1, and CA125. However, the contents of CEA, CYFRA21-1, and CA125 were decreased after 1 month or 3 months of treatment, and the observation group was lower than the control group (*P* < 0.05).

### 3.4. Comparison of T Lymphocyte Subsets between the Two Groups

As exhibited in Table 4, there was no significant difference in T lymphocyte subsets between the two groups before treatment (*P* > 0.05). After 1 and 3 months of treatment, CD3+ and CD4+/CD8+ in the two groups were higher than before, and the observation group was higher than the control group (*P* < 0.05). CD8+ in the two groups showed no significant difference after 1 and 3 months of treatment (*P* > 0.05).

### 3.5. Comparison of Serum IGF-1R and S100A2 Levels between Two Groups

Before treatment, there was no significant difference in serum IGF-1R and S100A2 levels between the two groups (*P* > 0.05). After 1 month and 3 months of treatment, serum IGF-1R and S100A2 levels in the two groups were higher than those before treatment, and the observation group was higher than the control group (*P* < 0.05), as shown in Table 5.

### 3.6. Comparison of the Incidence of Toxic and Side Effects between the Two Groups

Compared with the control group, there was no significant difference in the incidence of neutropenia, thrombocytopenia, and gastrointestinal reactions in the observation group (*P* > 0.05) (Table 6).

### 3.7. Long-Term Efficacy

One-year follow-up, disease progression time: the observation group was 129.85 days, and the control group was 89.74 days; half-year survival rate: the observation group was 98.00% (49/50), and the control group was 81.63% (40/49); 1-year survival rate: 76.00% (38/50) in the observation group and 53.06% (26/49) in the control group. The half-year survival rate and 1-year survival rate of the observation group were higher than those of the control group (*χ*^2^1 = 7.301, *χ*^2^2 = 5.698, both *P* < 0.05) (note: cases lost to follow-up have been excluded).

## 4. Discussion

Recently, particle implantation has been applied in the treatment of locally advanced cancer, in order to remit clinical symptoms, prolong survival time, and improve life quality of patients [5]. Dai et al. showed that the survival rates in 125I seed implantation treated-patients with III/IV NSCLC were significantly higher than those of conventional radiotherapy patients [6]. Another study confirmed that 125I seed implantation can effectively improve the disease control rate relative to conventional radiotherapy and chemotherapy in lung cancer patients [7]. 125I seed implantation is considered as an effective therapeutic option for patients with advanced lung cancer who have failed first-line chemotherapy [8, 9]. In view of this, the results showed that the disease remission rate was 41.18% with 125I seed implantation. It can be seen that although this radiotherapy has achieved certain curative effects in advanced lung cancer treatment, there is still room for improvement. Combining with other therapies to further enhance the antitumor effect is necessary.

BACE is an emerging method of local interventional therapy in recent years, in which chemotherapy drugs are directly infused into the supplying vessels of the lesions through catheters, and BACE is able to rise drug concentrations entering the lesions compared with superficial intravenous chemotherapy [10]. It has been reported that local therapeutic efficacy of BACE is 2-6 times that of intravenous chemotherapy [11]. BACE can maximize the therapeutic effect with a relatively small amount of chemotherapeutic drugs [12]. This work then investigated the use and the efficacy of BACE combined with 125I seed implantation in advanced NSCLC therapy based on the medical database. The results showed that the disease remission rate was higher in the observation group than that in the control group (62.75% *vs.* 41.18%). Compared with single 125I seed implantation, combined with BACE can significantly improve the antitumor effects. In addition, tumor markers are important indicators to reflect the occurrence, development, and prognosis of cancers. CA125, CYFRA21-1, and CEA are common clinical tumor markers. CYFRA21-1 is mainly distributed in lung tissue, and the concentration of CYFRA21-1 is significantly increased in NSCLC patients. Li et al. displayed that CA125 level was elevated in lung cancer patients and possessed a diagnostic sensitivity of more than 90% for lung cancer [13]. Previously, CEA is used to detect non-organ-specific tumor antigens, while study has revealed that CEA can be synthesized and released in lung cancer cells, and its concentration was linked with cancer recurrence, invasion, and metastasis [14]. This study showed that the serum levels of CYFRA21-1, CEA, and CA125 were lower after 1 month or 3 months of treatment both in two groups, indicating that both 125I seed implantation and the combined regimen of BACE and 125I seed implantation could achieve the purpose of anticancer. What is more, we also found that levels of cancer markers CYFRA21-1, CEA, and CA125 were much lower in the observation group than in the control group, implying that the combined regimen of BACE and 125I seed implantation, the direct injection of 125I into the lesions, can significantly improve the drug's ability to kill tumor cells and imped disease progression. Embolization with special materials could effectively block cancer blood supply and further enhance the anticancer functions [15].

Immunosuppression is prevalent in cancer patients, manifested by the abnormal function and disproportion of lymphocyte subsets, resulting in cancer cells successfully escaping immune surveillance of the host [16]. Step-by-step radiotherapy and chemotherapy have killing effects on T lymphocytes and normal tissue cells when killing cancer cells [17]. 125I seed implantation under the guidance of TPS system can advance accurate and precise radiation range; in addition to ensure the effective radiation dose in cancer target area, the damage to surrounding organs and tissues is small, which is beneficial to improve immune function of the body [9]. Besides that, BACE, as a local interventional chemotherapy, injects chemotherapeutic drugs into the lesion through a microcatheter and embolizes the target vessel with gelatin sponge; in addition to achieve antitumor effect, BACE has little influence on T lymphocytes and normal tissue cells and can effectively regulate immunity while inhibiting tumor growth [18]. In our study, the observation group showed higher levels of CD3+ and CD4+/CD8+ after 1 month or 3 months of treatment, suggesting that the combined regimen has a significant effect in regulating immunosuppression, which may also be the important mechanisms for the effectiveness of advanced lung cancer. IGF-1R was reported to have role as a multifunctional cell proliferation control factor, and the deregulated IGF-1R was correlated with the malignant differentiation and metastasis of lung cancer [19]. S100A2 was closely linked with the outcome of various malignancies, like lung cancer and breast cancer [20, 21]. In this study, the observation group exhibited lower serum IGF-1R level and higher serum S100A2 level after 1 month and 3 months of treatment. Patients in the observation group had a better half-year survival rate and 1-year survival rate. Therefore, we concluded that BACE combined with 125I seed implantation based on medical database could effectively improve the long-term efficacy of patients with advanced NSCLC by affecting the expression of IGF-1R and S100A2, as well as the immune system. In addition, this study also analyzed drug safety. The results showed combined regimen could not enhance the incidence of adverse reactions. The reason is considered that the continuous low-dose rate radiation treatment of radioactive particles combined with BACE can greatly reduce the systemic circulation drug dose and repress the genesis of adverse reactions and subsequently ensure the safety of patients. However, analysis using a larger cohort of the patients with NSCLC is essential to verify this conclusion.

In conclusion, BACE combined with 125I seed implantation based on medical database in the therapy of advanced NSCLC showed much stronger anticancer effects and could prolong the survival period and improve the survival rate.

## Figures and Tables

**Table 1:** Comparison of general information.

Project	Observation group (*n* = 51)	Control group (*n* = 51)	*t*/*χ*^2^
Gender (male/female)	27/24	30/21	0.358
Age (year)	40~85 (61.89 ± 7.10)	38~83 (63.02 ± 8.33)	0.737
Pathological classification			0.367
Squamous carcinoma	29 (56.86%)	32 (62.75%)	
Adenocarcinoma	22 (43.14%)	19 (37.25%)	
Clinical stage			0.354
IIIb	28 (54.90%)	25 (49.02%)	
IV	23 (45.10%)	26 (50.98%)	
Medical payment methods			1.221
Medical insurance	45 (88.24%)	49 (96.08%)	
Self-financed	6 (11.76%)	2 (3.92%)	

**Table 2:** Comparison of clinical efficacy between the two groups.

Group	Cases (*n*)	Complete remission (%)	Partial remission (%)	Stable (%)	Progress (%)	Disease remission rate (%)
Observation group	51	5 (9.80)	27 (52.94)	18 (35.29)	1 (1.96)	32 (62.75)
Control group	51	2 (3.92)	19 (37.25)	24 (47.06)	6 (11.67)	21 (41.18)
*χ* ^2^						4.752
*P*						0.029

**Table 3:** Comparison of tumor markers between the two groups.

Index	Group	Cases	Before treatment	After 1 month of treatment	After 3 months of treatment
CEA (mg/ml)	Observation group	51	62.35 ± 8.96	39.25 ± 6.48^a^	12.36 ± 3.28^a^
	Control group	51	64.01 ± 9.87	48.62 ± 7.12^a^	23.21 ± 5.46^a^
	*t*		0.889	6.951	12.165
	*P*		0.376	<0.001	<0.001
CYFRA21-1 (ng/l)	Observation group	51	8.24 ± 1.65^a^	6.15 ± 1.23^a^	3.65 ± 0.89^a^
	Control group	51	7.67 ± 1.52^a^	6.84 ± 1.10^a^	5.12 ± 1.00^a^
	*t*		1.815	2.986	7.842
	*P*		0.073	0.004	<0.001
CA125 (U/ml)	Observation group	51	27.96 ± 5.10^a^	22.36 ± 3.25^a^	12.96 ± 2.59^a^
	Control group	51	29.02 ± 5.69^a^	26.12 ± 3.78^a^	19.34 ± 3.51^a^
	*t*		0.991	5.386	10.445
	*P*		0.324	<0.001	<0.001

Note: compared with the same group before treatment, ^a^*P* < 0.05.

**Table 4:** Comparison of T lymphocyte subpopulations between the two groups.

Index	Group	Cases	Before treatment	After 1 month of treatment	After 3 months of treatment
CD3+ (%)	Observation group	51	55.32 ± 5.15	66.75 ± 5.69^a^	73.68 ± 6.98^a^
	Control group	51	54.72 ± 4.98	60.24 ± 5.33^a^	68.52 ± 5.70^a^
	*t*		0.598	5.954	5.301
	*P*		0.551	<0.001	<0.001
CD8+ (%)	Observation group	51	24.63 ± 4.31	24.12 ± 4.65	25.01 ± 5.25
	Control group	51	24.10 ± 4.10	24.35 ± 4.33	24.54 ± 4.87
	*t*		0.636	0.259	0.469
	*P*		0.526	0.797	0.640
CD4+/CD8+ (%)	Observation group	51	1.05 ± 0.29	1.41 ± 0.25^a^	1.55 ± 0.22^a^
	Control group	51	1.03 ± 0.25	1.22 ± 0.30^a^	1.34 ± 0.20^a^
	*t*		0.373	3.475	5.044
	*P*		0.710	0.001	<0.001

Note: compared with the same group before treatment, ^a^*P* < 0.05.

**Table 5:** Comparison of serum IGF-1R and S100A2 levels between the two groups.

Index	Group	Cases	Before treatment	After 1 month of treatment	After 3 months of treatment
IGF-1R (pg/ml)	Observation group	51	748.32 ± 68.52	672.35 ± 56.19^a^	612.52 ± 48.24^a^
	Control group	51	735.74 ± 72.69	704.64 ± 51.28^a^	675.58 ± 53.14^a^
	*t*		0.899	3.031	6.275
	*P*		0.371	0.003	<0.001
S100A2 (ng/ml)	Observation group	51	132.63 ± 20.29	174.62 ± 19.85^a^	198.59 ± 24.17^a^
	Control group	51	135.10 ± 23.74	160.02 ± 21.64^a^	169.78 ± 23.41^a^
	*t*		0.565	3.551	6.115
	*P*		0.574	<0.001	<0.001

Note: compared with the same group before treatment, ^a^*P* < 0.05.

**Table 6:** Comparison of the incidence of toxic and side effects between the two groups.

Toxic side effects	Group	Cases	I (%)	II (%)	III (%)	IV (%)	Total incidence (%)
Neutropenia	Observation group	51	8 (15.69)	5 (9.80)	0 (0.00)	0 (0.00)	13 (25.49)
	Control group	51	7 (13.73)	3 (5.88)	0 (0.00)	0 (0.00)	10 (19.61)
	*χ* ^2^						0.505
	*P*						0.477
Thrombocytopenia	Observation group	51	9 (17.65)	6 (11.76)	1 (1.96)	0 (0.00)	16 (31.37)
	Control group	51	5 (9.80)	8 (15.69)	0 (0.00)	0 (0.00)	13 (25.49)
	*χ* ^2^						0.434
	*P*						0.510
Gastrointestinal reactions	Observation group	51	6 (11.76)	4 (7.84)	1 (7.96)	0 (0.00)	11 (21.57)
	Control group	51	5 (9.80)	5 (9.80)	0 (0.00)	0 (0.00)	10 (19.61)
	*χ* ^2^						0.060
	*P*						0.807

Note: compared with the same group before treatment.

## Data Availability

The labeled dataset used to support the findings of this study is available from the corresponding author upon request.

## References

[1] Jonna S., Subramaniam D. S. (2019). Molecular diagnostics and targeted therapies in non-small cell lung cancer (NSCLC): an update. *Discovery Medicine*.

[2] Herbst R. S., Morgensztern D., Boshoff C. (2018). The biology and management of non-small cell lung cancer. *Nature*.

[3] Lu W., Du P., Yang C. (2018). The effect of computed tomography-guided^125^I radioactive particle implantation in treating cancer and its pain. *Cancer Biotherapy & Radiopharmaceuticals*.

[4] Zeng Y. W., Liu Y., Qi Y. (2021). Bronchial arterial infusion chemotherapy plus drug-eluting bead chemoembolization for recurrence of carina region-induced severe right main bronchial stenosis after pneumonectomy. *Clinical Lung Cancer*.

[5] Zhang J., Wu N., Lian Z. (2017). The combined antitumor effects of^125^I radioactive particle implantation and cytokine-induced killer cell therapy on xenograft hepatocellular carcinoma in a mouse model. *Technology in Cancer Research & Treatment*.

[6] Dai F., Wang J., An H. (2019). Therapy of ^125^I particles implantation inhibited the local growth of advanced non-small cell lung cancer: a retrospective clinical study. *American Journal of Translational Research*.

[7] Zhao G. S., Liu S., Yang L. (2020). Evaluation of radioactive 125I seed implantation for the treatment of refractory malignant tumours based on a CT-guided 3D template-assisted technique: efficacy and safety. *BMC Cancer*.

[8] Li C., Yao L., Gong J. (2020). Efficacy of gefitinib combined with 125I radioactive particles in the treatment of transplanted lung cancer tumors in nude mice. *Cardiovascular and Interventional Radiology*.

[9] Li W., Zheng Y., Li Y. (2017). Effectiveness of 125I seed implantation in the treatment of non-small cell lung cancer during R2 resection. *Oncology Letters*.

[10] Tezuka T., Inayama M., Suzue R., Miyamoto K., Haku T. (2020). A tuberculous bronchial artery aneurysm with abnormal findings on autofluorescence imaging bronchoscopy. *Internal medicine*.

[11] Lee H. N., Park H. S., Hyun D. (2021). Combined therapy with bronchial artery embolization and tranexamic acid for hemoptysis. *Acta Radiologica*.

[12] Boas F. E., Kemeny N. E., Sofocleous C. T. (2021). Bronchial or pulmonary artery chemoembolization for unresectable and unablatable lung metastases: a phase I clinical trial. *Radiology*.

[13] Li Z., Zhao J. (2021). Clinical efficacy and safety of crizotinib and alectinib in ALK-positive non-small cell lung cancer treatment and predictive value of CEA and CA125 for treatment efficacy. *American Journal of Translational Research*.

[14] Zhang Y., Huang J., Zou Q. (2020). Methylated PTGER4 is better than CA125, CEA, Cyfra211 and NSE as a therapeutic response assessment marker in stage IV lung cancer. *Oncology Letters*.

[15] Xiaobing L., Meipan Y., Pengfei X. (2022). Bronchial artery chemoembolization for hemoptysis in advanced primary lung cancer. *Clinical Lung Cancer*.

[16] van der Leun A. M., Thommen D. S., Schumacher T. N. (2020). CD8^+^ T cell states in human cancer: insights from single-cell analysis. *Nature Reviews Cancer*.

[17] Wang Q., Li S., Qiao S., Zheng Z., Duan X., Zhu X. (2021). Changes in T lymphocyte subsets in different tumors before and after radiotherapy: a meta-analysis. *Frontiers in Immunology*.

[18] Shang B., Li J., Wang X. (2020). Clinical effect of bronchial arterial infusion chemotherapy and CalliSpheres drug-eluting beads in patients with stage II–IV lung cancer: a prospective cohort study. *Thoracic cancer*.

[19] Wang R., Yamada T., Kita K. (2020). Transient IGF-1R inhibition combined with osimertinib eradicates AXL-low expressing *EGFR* mutated lung cancer. *Nature Communications*.

[20] Wang H., Zhang Z., Li R. (2005). Overexpression of S100A2 protein as a prognostic marker for patients with stage I non small cell lung cancer. *International Journal of Cancer*.

[21] Golouh R., Cufer T., Sadikov A. (2008). The prognostic value of Stathmin-1, S100A2, and SYK proteins in ER-positive primary breast cancer patients treated with adjuvant tamoxifen monotherapy: an immunohistochemical study. *Breast Cancer Research and Treatment*.

